# The Construction of an Action-Speech Feature-Based School Violence Recognition Algorithm and Occupational Therapy Education Model for Adolescents

**DOI:** 10.1155/2022/1723736

**Published:** 2022-05-27

**Authors:** Shuaiqing Zhang, Huan Li

**Affiliations:** ^1^Institute of Education, Joongbu University, Daejeon 32713, Republic of Korea; ^2^Education School, Fuyang Normal University, Fuyang, Anhui 236037, China

## Abstract

This paper constructs an algorithm for youth school violence recognition and an occupational therapy education model for victims through the extraction of action speech features. For the characteristics of violent actions and daily actions, action features in time and frequency domains are extracted and action categories are recognized by BP neural network; for complex actions, it is proposed to decompose complex actions into basic actions to improve the recognition rate; then, LDA dimensionality reduction algorithm is introduced for the problem of the high complexity of algorithm due to high dimensionality of features, and the feature dimensionality is reduced to 8 dimensions by LDA dimensionality reduction algorithm, which reduces the system running time by about 51% and improves the accuracy of violent action recognition by 3.3% while ensuring the overall performance of the system. The LDA dimensionality reduction algorithm reduces the number of features to 8 dimensions, which reduces the running time of the system by 51%, increases the accuracy rate of violent action recognition by 3.3%, and increases the recall rate of violent action recognition by 8.86% while ensuring the overall performance of the system. Based on the classical D-S theory, we proposed an improved D-S evidence fusion algorithm by modifying the original evidence model with a new probability distribution function and constructing new fusion rules, which can solve the fusion conflict problem well. The recall rate for violent actions is increased to 90.0%, thus reducing the missed alarm rate of the system.

## 1. Introduction

With increasing media coverage, the phenomenon of school violence has gradually come to the forefront of people's minds. With the development of the Internet, students on campus are exposed to all kinds of information from society, including violence and vulgarity [1]. Some students, out of curiosity, imitate the behaviors they see on the Internet, making the phenomenon of school violence more serious than ever. Teenagers need proper guidance and education during their formative years. However, school teachers and parents are unable to keep an eye on students, and those who are subjected to violence are often too afraid or shy to report it to teachers and parents promptly [2]. As a result, violence is not nipped in the bud at the earliest stages of its occurrence, and as a result, it grows worse and worse, seriously affecting the physical and mental health of the victim.

In recent years, there has been a growing trend of school violence in elementary and secondary schools, as reported by the news media. Minor forms of school violence include verbal abuse, pushing, and shoving, while severe forms of school violence include beating and abuse [3]. A domestic survey showed that, contrary to the perception of a stable school environment, more than 40 percent of students have experienced varying degrees of school bullying. Overseas, a 2010 USA Today survey reported that 50% of high school students surveyed had bullied others in the past year, 47% said they had been bullied, teased, or taunted, and 44% of boys and 50% of girls said they had been victims of school bullying [4]. This shows that bullying in schools is a very common and serious problem. Violence in schools jeopardizes the normal school and life of the victims and, more seriously, affects their worldview and outlook on life during their formative years. However, the victims of violent bullying are often afraid to give timely feedback to teachers and parents due to fear and self-esteem, thus causing the bullying children to be unable to be reassured and protected on the one hand, and the bullies are not promptly educated and supervised on the other, which eventually makes the phenomenon of school bullying increasingly serious.

A common problem in many school violence cases in recent years is that the bullied students are afraid to inform their parents or teachers about the bullying because they are afraid or threatened, thus causing an indelible psychological shadow on the children's young minds; in addition, the fact that violent incidents are not revealed leads to the perpetrators becoming increasingly rampant, which is also an important factor leading to the increase of school violence [5]. It is in this context that research on the active detection of violence in schools has emerged. Currently, smartphones are arguably the most widely used wearable sensor devices in the world, which include camera sensors (cameras), GPS sensors, proximity sensors, light sensors, inertial sensors (accelerometers and gyroscopes), and directional sensors (compasses). This topic is based on Video Data Detection of School Bullying aimed at achieving timely and proactive detection and reporting of school bullying by studying the identification of youth school violence based on action-voice features, using devices such as smartphones or bracelets to identify and analyze students' actions and detect the occurrence of violent actions [6].

## 2. Related Works

Foreign research on violent action detection was carried out relatively early, and the core problem of violent action recognition is to detect the target human action [7]. Some early researchers used the relevant features of sound to detect whether there is violence, and some researchers used a combination of video and audio and proposed a violent video detection model based on the semantic information corresponding to the audio and video data in the same video. O'Reilly et al. proposed the first video-based method to identify violent actions by detecting the presence of violence through the detection of blood and flames in images [8]. Menzies-Gow et al. proposed a violent action detection method using Lagrangian orientation fields to extract features from videos that are based on a spatiotemporal model using appearance, motion compensation of the background, and long-term dynamic information to ensure the scale of spatiotemporal features [9]. Feldstein et al. chose Gaussian Mixed Model (GMM) technique to extract the candidate regions where violent actions may occur from the information of optical flow and called suspicious activity [10]. Chen et al. propose to represent human behavior by a set of action units, and at the bottom, they propose a locally weighted word context descriptor to improve the traditional point-of-interest-based representation. This descriptor effectively incorporates neighborhood information [11]. At the high level, GNMF-based action units are introduced to bridge the semantic gap in action representation. León-Moreno et al. improve system robustness by fusing multisource heterogeneous sensor data, applying information fusion algorithms of fuzzy logic to recognize human behavior in fusion architectures, and performing feature layer fusion to improve recognition rates [12].

The frequent occurrence of school bullying has led to bad effects making school bullying an issue of widespread concern for the government and society [13]. Many studies have shown that school bullying is harmful to students for a long time, and as the research on school bullying deepens, school bullying, as a special type of comprehensive problem, is a very different concept from school violence, and domestic scholars have not yet formed a unified concept of school violence. The scholars Zhang et al. refer to school violence as an act in which students are physically and psychologically harmed in some way by teachers, classmates, and people from outside the school [14]. Li et al.'s view is that all acts of violence against teachers and students that occur within the school's authority are considered school violence [15]. Nickerson considers school violence to be all violent acts that students are subjected to, whether in public or private schools while attending school, participating in school activities, or after school. Professor Smith of the University of London's view on school bullying is that school bullying is a power struggle, where the strength of the stronger party often can bully and oppress the weaker party, and the bully is usually outnumbered and oppressed repeatedly, with a power mismatch [16]. Aiming at the problem that the recognition results of different parts of the sensor are seriously conflicting, the optimal fusion is carried out, and an improved D-S theory is proposed for fusion.

The research results on the definition of school bullying and the governance of school bullying at home and abroad are important academic resources for scholars at home and abroad to govern the social problem of school bullying from their different research perspectives, and they are also indispensable theoretical guidance for the practice of school bullying prevention and play an important role in practice [17]. However, it is easy to find from the literature review that the definition and prevention governance of school bullying emphasizes the legal obligations of the bully and the bullied, psychological construction, and regulations set by the state, while insufficient attention has been paid to the perspective of the motivation of bullying by school bullying subjects to produce school bullying behavior. To address adolescent school violence, this paper focuses on both the perpetrator and the victim and provides occupational therapy education to reduce the likelihood of school violence and its harmfulness.

## 3. Method

### 3.1. Research Design

Construction of an action speech feature-based school violence recognition algorithm and occupational therapy education model for adolescents, whose main research process is to collect human action data by wearing sensors such as accelerometers and gyroscopes on different parts of the body, after which the data are processed and fused and features are extracted to classify and identify school violence actions and give feedback to schools and parents, and the school, family, and society will work together to prevent and stop violence in schools.

The first step is to collect actionable data and preprocess them. Scenario simulation and data for the problem of school violence. This thesis is specifically for this scenario on campus, so as to simulate the campus environment more realistically. Together with the members of the project team, I conducted the experimental data collection for the campus violence scenario. The scenario experiment process included both daily campus actions such as running, jumping, and playing, as well as violent actions such as beating, pushing, and pushing down. Through multiple performances and rehearsals, the campus scenes were realistically restored and motion sensors and voice data were collected.

The second is the study of action feature extraction and feature selection algorithms. Feature extraction is one of the most important processes of pattern recognition and the process that has the greatest impact on recognition rate [18]. Before extracting the data, preprocessing of the data must be performed. The preprocessing part includes denoising of the received signal and real-time data segmentation. With the same data, different ways of action modeling can correspond to different numbers and types of features, so it is a research challenge to efficiently represent actions with fewer features. The extraction of action features lies in building appropriate action models on the one hand, and on the other hand, filtering and dimensionality reduction of the extracted high-dimensional features is also the key to reducing the complexity of the algorithm. The performance of action recognition based on a single part sensor is obviously inferior to that of multisensor fusion recognition, because multisensors can achieve a more comprehensive capture of actions, and the recognition performance can be improved by fusing different parts. In this paper, the relevant features are extracted in the time domain and frequency domain, and the basic useless features are initially eliminated by using the quadratic box plot method, and then, an improved Relief-F algorithm based on Filter is proposed for feature selection.

The third one is school violence recognition. The BP neural network classifier used in this paper learns through continuous feedback to determine the weights of nodes within different implicit layers and performs several classifier parameters' tuning and training method modifications to complete the classifier design work. For the problem of confusion between violent school actions and daily behavioral actions, a design scheme of joint action-speech feature recognition is proposed.

The fourth is a tripartite school-family-society effort, with schools and families avoiding and reducing the occurrence of school violence and, for those that have occurred, social occupational therapy and educational institutions providing professional psychological treatment for perpetrators and victims to reduce the damaging nature and after-effects of school violence on youth and society. In addition to physical training students, normal adult males can also be used as the subjects of this experiment. To match the theme of youth school violence in the article and fully tap the hidden information of school violence, the second-year physical training students of middle school are the most suitable group.

### 3.2. Participants

Scenario simulation and data for the campus violence problem. This thesis is specifically aimed at this scenario on campus, so as to simulate the campus environment more realistically. In this paper, through the recruitment of volunteers, 20 physical training students were recruited as participants in this experiment in the second grade of X middle school and randomly combined in groups of 10 people, named group A and group B, respectively.

The rationale for the selection of second-year physical training students from secondary school X in this paper is as follows.

1. Both age and physical characteristics were perfectly matched to the adolescent school violence perpetrators and victims
2. Physical training students are solid in all aspects of physical fitness due to years of sports training. They can very well complete the daily running, jumping, playing, and other campus action at the same time, complete the beating, pushing, and pushing down, and another violent action is not easy to be injured, and can ensure the maximum physical safety of the experimental participants
3. The second year of middle school is a critical time in the formation of life and values, and this age group is most likely to be involved in school violence

### 3.3. Measures

#### 3.3.1. Data Accounting Aspects

The number of network layers and the number of neurons were set for the neural network using the filtered and dimensionality-reduced features as the input to the neural network [19]. The transfer functions used in the implicit and output layers were determined after several trials. After that, we added the “fall” and “push” actions and reselected the features to determine the relevant parameters of the neural network. To address the problem that “hitting” actions are easily confused with nonviolent actions, the “hitting” actions were decomposed, and the data collection experiments of the decomposed actions were carried out to analyze the data and make the classification.

#### 3.3.2. Action Speech Recognition Aspects

Speech and action features are combined to further improve the action recognition rate. Firstly, the theory related to MFCC (Mel Frequency Cepstrum Coefficient) coefficients, which are very important in speech features, is introduced, and the MFCC and short-time energy features are extracted and classified for the speech data collected in the action test, and the results show that the classification effect of speech-based violence is much lower than that of motion sensor-based classification. Out of curiosity, some students imitated behaviors seen on the Internet, making the phenomenon of school violence more serious than ever.

#### 3.3.3. System Optimization Aspects

To optimize the built system, firstly, for the high time complexity of the system due to the excessive number of selected feature dimensions, the system is optimized by combining the dimensionality reduction algorithm to reduce the number of feature dimensions, which significantly reduces the recognition time of the system and lays the foundation for future hardware implementation. In addition, the problem of serious conflicts between the recognition results of different parts of the sensor is optimized fusion and proposed to improve the D-S theory for fusion, simulation analysis, and adaptive adjustment of the decision layer class fusion algorithm for comparison and analysis of the conclusions.

### 3.4. Design

The study is based on multisensor fusion recognition, so the location and number of sensors are crucial. The study shows that the built-in sensors of wearable devices are located in different locations, and the number of sensors will have a direct impact on the recognition results. For different actions, different locations of sensors will have different recognition accuracy [20]. At present, most of the recognition of human actions are located at the waist, legs, wrists, and chest; in addition, for the fusion recognition system of multiple sensors, there are still multiple choices of combinations of different locations. “Lying,” “sitting,” “standing,” “walking,” “running,” “going upstairs,” “going downstairs,” “jogging,” “jumping,” and other daily movements, the current common positions, and combinations of study results in specific performance comparisons are shown in Table 1. Through comparison, it can be found that the performance of action recognition based on a single part sensor is inferior to multisensor fusion recognition, which is because multisensor can achieve more comprehensive capture of action, and fusing different parts can improve recognition performance. In addition, the combination of different parts has a greater impact on recognition accuracy, and research shows that the more sensors are not the higher the recognition accuracy, and the number of sensors worn needs to consider the balance of convenience and recognition rate. In this project, the data was collected by wearing sensors on the waist, legs, and wrists, and combined with the current research, it was decided to use the sensors on the waist and legs for fusion detection of violent campus movements. Therefore, in this study, the motion sensor was placed on the waist of the experimenter, and the triaxial acceleration and triaxial gyroscope signals were collected.

The action recognition system mainly consists of the following parts: data acquisition and processing, feature extraction and selection, and classifier design. At present, the common idea of data segmentation is to set a sliding window, and the data collected by the sensor is stored in the form of the data stream, by choosing a suitable window length, sliding in the time axis of the data stream according to a certain ratio and speed can be. In this paper, the window length is set to 256 sampling points, and the sampling frequency of the collected data sensor is set to 50 Hz, so the time length of each extraction is about 5 s. After comparison, the data within this time length can fully reflect the change of action and can meet the requirements of final recognition. In addition, since the feature extraction needs to be analyzed in the frequency domain afterward, the design length of the sliding window is chosen as a power of 2 for the convenience of time-frequency conversion.

Victims of violence often do not dare to report the situation to teachers and parents in a timely manner out of fear or shyness. This leads to the fact that in the early stages of violence, violence cannot be nipped in the bud. BP neural networks are no longer suitable for places with high real-time requirements due to their global approximation nature and thus very slow learning speed, and the deep learning-based Convolution Neural Network (CNN) has the advantages of no manual feature selection and excellent classification effect, but the training network requires a large amount of sample data, which is very demanding for equipment performance requirements are very high. Compared with BP and Convolutional Neural Network, Radial Basis Function (RBF) has the advantages of simple network structure, fast convergence, and the ability to fit any nonlinear function, so it is widely used in various fields [21].

Since the acquisition of action data is affected by many noises, for this reason, it is necessary to choose a suitable method for smoothing and denoising. Several commonly used filtering and denoising methods are mean, median, smoothing, Gaussian, and low-pass. Among them, smoothing filtering is easy to operate and simple to understand. In a segment of data, the average of the neighboring points is sought, and the size of its selected neighborhood cannot be too large; otherwise, it will produce information loss. Median filtering is to select the middle value to avoid the influence of noise, which will not produce edge information loss, simple calculation, and is easy to implement with hardware. Mean filtering replaces the average value of multiple points around a point with a small number of points that will have large fluctuations in the average value. Gaussian filtering is replaced with a weighted average of its own and the data in the field, yielding a broken flat edge problem. Low-pass filtering can be thought of as setting a fixed frequency above which the frequency domain is filtered out and vice versa, which is allowed to pass. Since the human body movement frequency is relatively small, the normal movement is between 1 and 50 Hz. Therefore, the IIR Butterworth (Butterworth) low-pass filter is selected to remove the noise, calculated as follows.

(1) $$\begin{array}{c} h\left({nT}_{s}\right)=g\left(t\right)+\underset{n=1}{\sum }\delta \left(t+nT\right). \end{array}$$

To make the processing of the collected data easier, the data is normalized. The data is scaled to make the data in a certain limited area. Normalization is a dimensionless processing method that makes the values relative and units the data with different ranges so that they have a uniform distribution and are easier to calculate and understand. The minimum-maximum normalization method of normalization, also known as discrete normalization, is used in this paper.

(2) $$\begin{array}{c} \sigma_{i}=\frac{1+u_{i}}{\max\left(u_{i}\right)+\min\left(u_{i}\right)}. \end{array}$$

Since each person completes an action with a different amplitude and frequency, the length of the data collected by the sensor is not the same, and it takes a relatively long time to collect action and accumulate a large amount of data. For this reason, the collected data need to be regularized and segmented into different windows, with adjacent windows partially overlapping, and the features of the windows are extracted to provide an accurate description of the human action characteristics. Three common window addition methods are sliding window segmentation, event-based definition window segmentation, and action-based window segmentation.

(3) $$\begin{array}{c} w\left(n\right)=\left\{\begin{array}{c} 0,n\leq N\left(N>=0\right),\\ 1,n>N\left(N>=0\right). \end{array}\right. \end{array}$$

The time length of each extraction is about 5 s. After comparison, the data within this time length can fully reflect the change of an action, which can meet the final identification requirements. For the input of the deep learning network, this section adopts the strategy of dividing the original audio waveform into frames and then using the corresponding waveform map of each frame as the input of the AlexNet network to extract the audio features of the original waveform. Finally, the audio features are fed into the LSTM network for modeling the timing signal. The output of the last LSTM unit is the memory of the most effective features of the whole audio segment, after which the FC layer is connected to classify the audio segment effectively. Block diagram of the violence audio detection system based on the original audio waveform is shown in Figure 1.

### 3.5. Analysis

The DS fusion algorithm, when faced with severely conflicting evidence, fuses the result as a violent event and ignores the credibility of voice evidence; the Yager fusion algorithm, when faced with severely conflicting evidence, synthesizes the result showing that the Yager fusion process reduces the credibility of both sets of evidence, and while assigning more support to the uncertainty function, i.e., it does not make an exact judgment, which is not applicable in practical scenarios. Compared with the improved Yager synthesis result, the proposed improved solution reduces the credibility of video evidence and increases the credibility of voice evidence, but the synthesis rule in this paper assigns conflicts to the focal elements that generate conflicts, while the improved Yager assigns conflicts to all focal elements. The improved Yager fusion algorithm is more reasonable than the improved Yager fusion algorithm. On the one hand, the bullied children cannot be comforted and protected, and on the other hand, the bullies have not received timely education and supervision, which eventually makes the phenomenon of school bullying increasingly serious.

In the network training process, we only need to train the parameters of the LSTM network since the parameters of the CNN (AlexNet) network that takes the features are trained. The maximum number of iterations is set to 100, and the loss value varies with the number of iterations. To characterize the envelope of the audio in the long-time range, we also take the statistical features. The violent audio detection method based on acoustic features and long-time statistical features achieves better detection results. In terms of deep learning, this paper adopts two strategies, original waveform as network input and audio speech spectrogram as network input, and after comparison, we find that the end-to-end detection method based on the original audio waveform is more beneficial to violent audio detection. This also provides a new idea for the later audio-video feature fusion method.

## 4. Results

The background of this study is for school violence scenarios, to truly simulate school violence actions to ensure the practicality of the recognition system, for complex violent actions through the protection measures to ensure that the data is real and reliable, and the use of several different experimental subjects to repeatedly simulate various types of actions, so that the collection database is more convincing. The collected actions include “hitting,” “pushing,” “pushing down,” and other common school violence actions and “running,” “playing,” and “jumping.” The first step is to identify these nine types of actions. These nine types of actions are identified, and finally, the performance indexes are measured according to violent and nonviolent actions. Not all the proposed features are useful for classification and recognition, after which they are firstly screened by using quadratic box plots to distinguish useless features for actions and then studied by using feature selection algorithms. A comparative study was conducted on two groups of physical training students, A and B. The test index data of the experimental group were analyzed by mathematical and statistical methods. The experimental results demonstrate that the fusion algorithm has improved the recognition rate of actions compared to any single part sensor, and the recognition rate is 85.3%, especially for violent actions after the fusion. The recognition rate of complex actions such as “fall,” “push,” “push,” and “hit” is improved by 7.2%. By calculating the four index parameters, we can see that the overall system performance is improved by about 4.98%. The solution will also be proposed for the fusion problem in the case of conflicting sensor recognition of different parts, to improve the recognition rate of complex actions such as “fall” and “push down.” In this paper, “push” and “fall” actions are added. However, the action process of fall is short, as shown in Figure 2, which shows the change of acceleration sensor during the occurrence of violent action.

### 4.1. Motion Speech Feature Extraction

A 5-fold cross-validation was used to test the performance of the model, and the test samples were divided into 5 equal parts, and the average of the 5 recognition results was taken as the result, and four metrics, accuracy, precision, recall, and F1-score, were selected to evaluate the classification algorithm. The test and evaluation results for the three audio databases are shown in Table 2.

Table 2 shows that the classification algorithm achieves a correct rate of 88.33% on the self-made speech database, the highest correct recognition rate of 95% on the Finnish speech database, and 91.67% on the CASIA public speech database, which indicates that the classification algorithm has a better performance in recognizing speech emotion. In addition, the recall rate on all three speech databases is above 85%, which indicates that the F1-score of the classification algorithm is the highest for the Finnish speech database, followed by the CASIA database, which indicates that the classification algorithm has the best performance on the Finnish speech database, followed by the CASIA database and the homemade speech database. The reason for the analysis is that for the home-made small speech database, the subject members had poor performance in expressing emotions through speech, which resulted in the difference between bullying emotions and nonbullying emotions not being obvious, which had an impact on the final correct recognition rate. However, the Finnish speech database is a school bullying and nonbullying scenario simulated by elementary school students, which is very suitable for the needs of this topic, so the classification algorithm performs best on this database. The CASIA speech database is recorded by professionals, and the emotions expressed by speech are fuller, and the differences in emotions expressed by different speech are larger, so the differences in feature vectors are also larger. The classification algorithm performs better on the Finnish speech database and the CASIA speech database.

In the experiment, 14 kinds of action data were collected for each person, and there were 20 people in total. 15 people's action data from each action were selected as training set samples, and 5 people's action data were selected as test set samples, and there were 210 samples in the training set and 70 samples in the prediction set. In the previous mathematical theoretical derivation, it has been found that the penalty factor and radial kernel function parameters are two important parameters for SVM classification performance. Therefore, this paper discusses the comparison of SVM classification performance after four random choices of these two parameters and after PSO parameter optimization (Figure 3). Radial Basis Function (RBF) network has the advantages of simple network structure, fast convergence speed, and the ability to fit arbitrary nonlinear functions, so it has been widely used in various fields. Comparison of SVM classification performance after PSO parameter optimization: the results of four times random parameter search under time-domain features have been compared with the SVM classification performance after the PSO parameter optimization process, and the range of random selection process *c* and *g* is (0,100). The random selection of different two important parameters directly affects the classification performance of the SVM. As the number of iterations increases, the red best-fit curve shows an increasing trend of classification recognition rate, which reaches the optimum and remains unchanged when it reaches 8 iterations, with an accuracy of 96.97% under fivefold crossover, a penalty factor *c* of 1.6294, and a radial kernel function *g* of 11.0116, and the SVM classification model is built with these two optimal parameters, which finally obtains a classification recognition rate of 92.85%.

### 4.2. Campus Violence Identification

In the conversion rate of violent action recognition, because the amplitude of motion is close to the interaction between violent action and running motion, to improve its action recognition accuracy, a method of joint recognition by multilayer classification algorithm should be designed, and then, the extracted features are analyzed and processed. Firstly, the SVM algorithm is used to recognize them, and then, the threshold decision tree classification algorithm is used in the decision layer to further classify the classification level. Finally, the two prediction results are combined and then weighted, the weights of the features are reasonably assigned, and finally, a DT-SVM multilayer classification model is established to improve the action recognition rate. Here, the selected features are first analyzed to find out the decision threshold of a certain type of action. Since some features with certain thresholds can directly distinguish violent and nonviolent behaviors, for example, the spacing of the center of mass and the magnitude of the action, the probability of nonviolent behaviors can be directly determined when there is no obvious action in the video and the active participants are very far away, or the probability of violent behaviors is significantly increased when one of the action participants falls. In this paper, relevant features are extracted in the time domain and frequency domain, respectively, and the basic useless features are initially eliminated by the quartile box plot method, and then, an improved Relief-F algorithm based on Filter is proposed for feature selection. On the premise of the recognition rate, the feature dimension is reduced by the dimensionality reduction algorithm for system optimization.

A total of 12448 violent action frames, 9963 nonviolent action video frames, and 2485 nonviolent undetected target video frames were collected. A total of 17 features were extracted, and the feature selection algorithm was used to select the optimal parameters after filtering the features and thresholds for recognition using fivefold cross-validation. The results show that 96.52% of violent actions are accurately identified as violent actions, and 3.48% are incorrectly identified as nonviolent actions. 80.81% of nonviolent actions are accurately identified as nonviolent actions, and 19.19% of nonviolent actions are incorrectly identified as violent actions. The final obtained classification accuracy using only the SVM classification algorithm was 89.54%, accuracy was 94.90%, the recall was 80.81%, and algorithm performance parameter F1_S was 87.29%. As shown in Figure 4, compared to the DT-SVM algorithm with only the inclusion of video frames with obvious actions, the DT-SVM algorithm with the inclusion of some undetected target frames has 0.78% higher accuracy, 2.14% higher precision, 0.74% higher recall, and 1.31% higher algorithm performance. The undetected target frames can be detected well in the foreground detection stage, and the partial undetected target frames are added only to demonstrate the algorithm's classification of undetected target frames.

### 4.3. Constructs of Occupational Therapy Education Models

Studies have found that the development of adolescent personality is closely related to family education and living environment. Children who lack parental companionship tend to be withdrawn and quiet. Especially children left behind, because their parents are not around, food, clothing, housing, and transportation are not well taken care of, and even when they are bullied, they have no place to cry because their parents are not around, and overall, they develop a withdrawn, introverted, and timid personality. In addition, without parents to “back up,” they are bullied and have no way to complain and gradually become victims of school violence.

In the rapidly developing economic era, most parents are only concerned with making money to support their families and believe that their children only need to study hard and have stable and excellent academic performance. Parents rarely participate in their children's growth process and lack the necessary communication with their children. Children increasingly reject open communication with their parents or fear communication with their parents, which may lead to certain psychological disorders. At the same time, parents' bad habits may also set the wrong values for their children, for example, parents often drink in front of their children and quarrel and fight with each other, and children will learn from their parents' bad habits and become violent over time. What is more, some parents lack of patience, and the child made a mistake, indiscriminately is a beating, and eventually, the child encountered anything also choose to save violence, and such children gradually become the perpetrators of school violence. To distinguish between school violence and daily actions, this paper designs an action-speech joint feature recognition model. The model is mainly designed to be equipped with sound-collecting sensors. Violence in schools is often accompanied by the bully's loud abuse and the victim's crying. And the large-scale movements such as running, jumping, and falling are not accompanied by insults and crying.

Middle school students are in early adolescence. Most adolescents are psychologically adventurous and impulsive, and they like to imitate others' words, actions, and dresses. Most adolescents are adventurous and impulsive, and they like to imitate others' words, behaviors, and dresses. This period of adolescence is accompanied by many shortcomings, such as more contact with social things but lack of social experience, relatively reckless and lack of rational thinking and even reckless to achieve some immature purposes, weak ability to distinguish right from wrong, and easily influenced by the negative environment around them and the violent factors in movies and online games. If we do not control and guide them correctly, they will easily go astray and do things that are detrimental to their good development and even endanger social security in serious cases.

Different from previous studies that focused unilaterally on victims of school violence, this paper analyzes the psychological factors of both perpetrators and victims and constructs a perpetrator-victim occupational therapy education model for the different psychologies of perpetrators and victims, as shown in Figure 5.

In response to incidents of school violence that have occurred, schools, families, and society should act proactively and cooperate to provide reasonable psychological guidance to perpetrators and victims of violence to avoid lifelong psychological trauma.

*For the abuser*. Abusers themselves often have deficiencies in emotional communication and self-behavior control, such as a lack of proper emotional communication skills, empathy, and proper self-behavior control methods, leading them to find an outlet to vent and express themselves and eventually to take the path of bullying others. The important reason we need to pay attention to and take effective measures to help the bully improve their own words and behaviors is based on understanding and respecting each individual, guiding them to establish a correct sense of communication and interaction based on understanding the motivation of the bully's behavior, and providing some methods and skills to improve their own words and behaviors, so that the bully knows the harm of bullying others and that the bullying behavior can be corrected, and so that the bully will feel accepted, understood, and trusted and will then take the initiative to improve his or her behavior and speech.

*Targeting victims*. A generalized analysis of students' responses to violence on secondary school campuses shows that more than half of the victims chose to keep quiet after being subjected to violence on school campuses, and they chose to keep quiet because they were afraid of the abuser's reoccurrence. Very few of the victims were affected by the violence, but their normal school life was affected to a certain extent. Some students who are victims of campus violence have mental problems, such as fear and suspicion all day long, serious fear of the campus and the abuser, and are afraid to come to school. Some students even have a nervous breakdown and become mentally ill. Some students choose to end their lives to escape the violence. For victims of school violence, it is important to focus on psychological and emotional relief in addition to physical treatment. It is important to guide the victims to come out of the gloom, believe in society again, and work hard to live a positive life. It is also important to instill a sense of courage to speak out in the face of school violence. If violence occurs on campus, report it to the teacher first to receive appropriate assistance, and do not be reckless and retaliate against the perpetrator to vent your anger and prevent the violence from escalating again. It is best to avoid being alone on the way to and from school and to avoid choosing roads with few people and remote locations. When you go out alone, pay attention to strangers, do not meet with people you know online, and do not go to Internet cafes, game halls, and other entertainment places that you are not allowed to enter. In short, only by learning to protect yourself and having a strong sense of protection can you avoid being harmed by school violence.

## 5. Discussion

Usually, when the topic of school bullying is mentioned, people will express their opposition or hatred, putting the bully in the position of the weak and the bully in the position of the strong. However, both the bully and the bullied in school bullying incidents are in a vulnerable position, and neither of them uses the right ways or methods to express their emotions and needs and maintain their interpersonal relationships. The bullies themselves often have deficiencies in emotional communication and self-behavior control, such as a lack of proper emotional communication skills, empathy, and proper self-behavior control methods, resulting in their need to find an outlet to vent and express themselves and eventually taking the path of bullying others. The important reason why we should pay attention to and take effective measures to help bullies improve their own words and behaviors is based on understanding and respecting each individual, guiding them to establish a correct sense of communication and interaction based on understanding the motivation of the bully's behavior, and providing some methods and techniques to improve their own words and behaviors, so that the bully knows the harm of bullying others and that the bullying behavior can be corrected, so that the bully will feel accepted, understood, and trusted and will then actively participate in improving their speech and behavior, experience the positive effects of improving their speech and behavior, and then eliminate the bullying behavior.

## 6. Conclusion

In this paper, we studied the action characteristics of violent actions and collected data on “push,” “push down,” “squat,” and “roll.” The simulation shows that the average recognition accuracy is 88.35%, and the recall rate of violent action recognition is 84.63%. To address the feature redundancy problem of the Relief-F feature selection algorithm, a redundancy improvement algorithm is proposed, a multilayer classifier based on decision tree-RBF neural network is built, and a PACBF algorithm is designed for adaptive fusion processing in the decision layer. For the problem of fusion conflict of multipart recognition results, an improved D-S theoretical fusion model is proposed to modify the original evidence model by designing a new distribution function and constructing a new fusion rule, which finally achieves a system recognition rate of 93% and a recall rate of 91%, greatly reducing the system leakage rate. The occupational therapy model is theoretically able to address the negative effects of school violence on both perpetrators and victims, but due to time limitations, the selection of psychology professionals is not ideal, and the next work can be conducted in more detail and depth in this area.

## Figures and Tables

**Figure 1:** Block diagram of the violence audio detection system based on the original audio waveform.

**Figure 2:** Schematic diagram of acceleration sensor changes for fall-like movements.

**Figure 3:** PSO-SVM parameter search process in the time domain.

**Figure 4:** Quartile plot of *y*-axis variance characteristics of waist data.

**Figure 5:** Perpetrator-victim occupational therapy education model.

**Table 1:** Performance comparison of multisensor position combinations.

Sensor combination	Average recognition rate
Legs	83.57%
Waist	84.21%
Chest	80.01%
Legs+chest	82.17%
Legs+waist	91.46%
Chest+waist	91.09%
Waist+legs+chest	88.60%

**Table 2:** Speech emotion classification test results.

Voice library name	Accuracy	Precision	Recall	F1-score
Self-made voice library	88.10%	88.30%	94.80%	93.10%
Finland	94.80%	89.20%	95.40%	89.80%
CASIA	94.60%	87.50%	91.70%	89.60%
SMiN	87.40%	92.50%	89.70%	88.50%

## Data Availability

The data used to support the findings of this study are available from the corresponding author upon request.
